# Performance for rotor system of hybrid electromagnetic bearing and elastic foil gas bearing with dynamic characteristics analysis under deep learning

**DOI:** 10.1371/journal.pone.0244403

**Published:** 2021-03-15

**Authors:** Xiangxi Du, Yanhua Sun

**Affiliations:** School of Mechanical Engineering, Xi'an Jiao Tong University, Xi'an City, China; University College London, UNITED KINGDOM

## Abstract

The bearing-rotor system is prone to faults during operation, so it is necessary to analyze the dynamic characteristics of the bearing-rotor system to discuss the optimal structure of the convolutional neural network (CNN) in system fault detection and classification. The turbo expander is undertaken as the research object. Firstly, the hybrid magnetic bearing-rotor system is modeled into the form of four stiffness coefficients and four damping coefficients, so as to analyze and explain the dynamic characteristics of the system. Secondly, the ambient pressure is introduced to analyze the dynamic characteristics of the elastic foil gas bearing-rotor system based on the changes in the dynamic stiffness and dynamic damping of the gas bearing. Finally, the CNN is introduced to be applied in the detection of faults of bearing-rotor system through determining the parameters of the constructed CNN. The results show that the displacement of the rotor increases and the stiffness decreases with the acceleration of the speed of the electromagnetic bearing. The maximum displacement of the rotor can reach 135μm, and the maximum stiffness can be reduced to 35×10^5^N/m. Increase of ambient pressure causes enhancement of main stiffness of the gas bearing, and the main damping decreases accordingly. Analysis of the classification accuracy and loss function based on the CNN model shows that the convolution kernel size of 7*1 and the batch size of 128 can realize the best performance of CNN in fault classification. This provides a data support and reference for studying the dynamic characteristics of the bearing-rotor system and for the optimization of CNN structure in fault classification and detection.

## 1. Introduction

In equipment with high rotor speed such as turbo expander, it is difficult to meet the working requirements of the equipment only by relying on oil to lubricate the bearings. The emergence of magnetic bearing and gas bearing can solve such problem well. Of which, magnetic bearing is a kind of mechatronic product. By energizing the alternating current (AC) coil of the stator, electromagnetic force is generated between the stator and the rotor to realize the journey [1,2]; while the gas bearing uses gas as the lubricating medium, and the direct contact between the rotor and stator can be avoided through the formation of a gas film between the shaft and the bearing [3,4]. Currently, there are many researches on the magnetic bearing-rotor system and the foil gas bearing-rotor system. For example, Du et al. (2019) analysed the impacts of stiffness and damping changes on imbalance response of rotor by adjusting the stiffness targeting to uneven distribution of rotor mass caused by mechanical processing and assembly error; it was found that the bearing being farther away from the imbalance position has the larger rotor displacement and bearing load, and increase in stiffness and damping of active electromagnetic bearing will increase the load on the bearing, thereby reducing the response displacement of the rotor [5]. Fernando and Saha (2018) adopted the mechanical and electromagnetic finite element models to discuss the design scheme of the magnetic flux modulated dual rotor structure and the trade-off relationship among the weight, loss, and shear stress of the dual rotor structure [6]. Samanta et al. (2019) gave an overview of the development status of foil gas bearing technology and an in-depth discussion on the complexity related to the compressible flow geometry and the dynamic performance and stability related to stiffness and damping [7]. Bailey et al. al. (2018) completed the establishment of the gas-lubricated bearing coupling model starting from the extended dynamics system, and conducted an in-depth investigation on the impact of key bearing parameters on bearing dynamics [8].

Due to its excellent performance, deep learning methods have been applied in many fields [9]. Relevant experts and scholars have conducted corresponding researches to study its application in bearing-rotor system. Ma and Chu (2019) applied the convolutional residual networks (CRN), deep belief networks (DBN), and deep autoencoder methods (DAM) in the system, and taken multi-objective optimization algorithms as an integrated strategy to achieve effective diagnosis of rotor and bearing faults in rotating machinery [10]. Hoang and Kang (2019) gave a comprehensive review on the application of autoencoders, CNN, and restricted Boltzmann machines (RBM) in bearing fault diagnosis [11]. Udmale et al. (2019) proposed a fault classification intelligent diagnosis method based on deep learning kurtogram and sequence model (DPKS), and found that the method showed high classification accuracy in fault diagnosis [12]. Li et al. (2019) proposed an intelligent remaining service life prediction method based on deep learning for the degradation in the long-term operation [13]. Therefore, there has been a relatively large amount of research work on magnetic bearing and gas bearing, but there is relatively little research on the dynamic characteristics of bearing-rotor system. In addition, it still lacks the introduction of deep learning methods into research work in this field relatively.

To analyze and discuss the dynamic characteristics of magnetic bearing and gas bearing-rotor systems, and to analyze the applicability of CNN in detection of system fault, this article takes turbo expander as the research object and discusses the dynamic characteristics of hybrid magnetic bearing and elastic foil gas bearing-rotor system. It is a crucial innovative point of this article. This research aims to provide a data reference for the dynamic characteristics analysis of the bearing-rotor system and expand the application of deep learning methods in this field.

## 2. Methods

### 2.1 Working principles of rotor system of magnetic bearing and elastic foil gas bearing

From a functional point of view, both magnetic bearing and gas bearing are high-speed support means with their own unique characteristics [14,15]. Of which, the magnetic bearing uses electromagnetic force to enable the rotor to float in the space, which also enables no mechanical contact between the support and the supported component [16]. According to the different principles, it can be divided into three types: active, passive, and hybrid. This article mainly studies the performance of rotor system for hybrid magnetic bearing. The working principle of the magnetic bearing-rotor system is shown in Fig 1 below. Specifically, the magnetic levitation rotor can be suspended after power on. The main function of the displacement sensor is to detect the signal related to the rotor and the movement offset, and then transmit the detected related information to the controller. The main function of the controller is to use appropriate control algorithm tool to calculates and obtain the control signal, and the obtained control signal is converted into a control voltage or current after the power amplifier, so as to realize the control of the electromagnet. Finally, the rotor is adjusted to the balance position to achieve high-speed rotation [17].

**Fig 1:** Working principle of magnetic bearing-rotor system.

Different from magnetic bearing, foil gas bearing is a kind of dynamic pressure fluid lubrication bearing [18]. For foil gas bearing, the foil can give the bearing elastic support, which promotes the realization of the wedge effect between the rotor and the bearing. At the same time, the elastic foil can also provide the rotor with appropriate structural stiffness and damping, which can solve poor bearing capacity and poor damping caused by too large stiffness. The basic composition of elastic foil gas bearing is shown in Fig 2 below.

**Fig 2:** Basic composition of elastic foil gas bearing.

### 2.2 Dynamic characteristics of rotor systems for magnetic bearing and foil gas bearing

#### Hybrid magnetic bearing-rotor system

The hybrid magnetic bearing-rotor system and the foil gas bearing-rotor system in turbo expander are undertaken as examples. For the hybrid magnetic bearing, the fan wheels and working wheels with complex structures located at both ends of the bearing are replaced with discs with the same moment of inertia, and the bearing is modelled into an elastic damping support composed of four stiffness coefficients and four damping coefficients. The equation of motion corresponding to a hybrid magnetic bearing-rotor system with five degrees of freedom can be expressed as below:

$$\left[Q\right]\left\{\overset{¨}{X}\right\}+\left[D\right]\left\{\dot{X}\right\}+\left[R\right]\left\{X\right\}=\left\{F\right\}$$ (1)

In the above equation, [*Q*] represents the mass matrix, [*D*] represents the damping matrix, [*R*] represents the stiffness matrix, {*X*} refers to the generalized displacement vector, and {*F*} refers to the forced vibration force vector.

Thus, the motion equation of the hybrid magnetic bearing-rotor system under free vibration can be expressed as Eq (2) below.

$$\left[Q\right]\left\{\overset{¨}{X}\right\}+\left[D\right]\left\{\dot{X}\right\}+\left[R\right]\left\{X\right\}=0$$ (2)

In the hybrid magnetic bearing, if the rotor is in a stable state, then the rotor is at the axis position; if the system is subjected to external loads, it will cause the rotor to deviate; and it can result in stable suspension of rotor in the hybrid magnetic bearing through the coordinated action of the displacement sensor and the controller. To analyse the dynamic stability of the hybrid magnetic bearing-rotor system, the system is tested for multiple rounds through experiments, and the effects of the external load on the performance of the magnetic bearing-rotor system under a stable suspension state and different speeds are analysed to reveal the dynamic characteristics of the magnetic bearing.

#### Elastic foil gas bearing-rotor system

For the turbo expander, the air sucked by the fan is directly obtained from the atmosphere, and is directly discharged into the atmosphere after the required pressure is reached, which causes a waste of expander power [19]. For elastic foil gas bearing, the lubricating medium used is compressible fluid, and the flow pressure generated by this lubricating medium is closely related to the ambient pressure. Based on this, the fan wheel in the elastic foil gas bearing-rotor system is replaced with a pressurizer, and the pressurized gas is supplied to the foil gas bearing, so that the ambient pressure at the end of the foil bearing can be elevated. For this reason, the dynamic characteristics of the elastic foil gas bearing-rotor system are analysed from the ambient pressure. In addition, the influencing effects of ambient pressure on the critical rotating speed of elastic foil gas bearing-rotor system, dynamic stiffness and dynamic sampling of the foil gas bearing at different rotating speed are analysed to discuss the dynamic characteristics of the elastic foil gas bearing-rotor system. Of which, the equation expression and calculation of stiffness coefficient is given as below:

$$\left[\begin{array}{cc} S_{xx} & S_{xy}\\ S_{yx} & S_{yy} \end{array}\right]=\left[\begin{array}{cc} \frac{\partial F_{x}}{\partial x} & \frac{\partial F_{x}}{\partial y}\\ \frac{\partial F_{y}}{\partial x} & \frac{\partial F_{y}}{\partial y} \end{array}\right]=-\frac{r^{2}Pa}{c}\int_{-\frac{1}{2}}^{\frac{1}{2}}\int_{0}^{2\pi }\left[\begin{array}{cc} P_{x}\sin\;\theta & P_{y}\sin\;\theta \\ P_{x}\cos\;\theta & P_{y}\cos\;\theta \end{array}\right]d\theta d\xi$$ (3)

Damping coefficient *D* can be calculated with below equation:

$$\left[\begin{array}{cc} D_{xx} & D_{xy}\\ D_{yx} & D_{yy} \end{array}\right]=\left[\begin{array}{cc} \frac{\partial F_{x}}{\partial \dot{x}} & \frac{\partial F_{x}}{\partial \dot{y}}\\ \frac{\partial F_{y}}{\partial \dot{x}} & \frac{\partial F_{y}}{\partial \dot{y}} \end{array}\right]=-\frac{r^{2}Pa}{c}\int_{-\frac{1}{2}}^{\frac{1}{2}}\int_{0}^{2\pi }\left[\begin{array}{cc} P_{{}_{x}}^{\prime }\sin\;\theta & P_{{}_{y}}^{\prime }\sin\;\theta \\ P_{{}_{x}}^{\prime }\cos\;\theta & P_{{}_{y}}^{\prime }\cos\;\theta \end{array}\right]d\theta d\xi$$ (4)

In the above two equations, *P* is the pressure, *F* refers to the vector force, *r* refers to the rotor radius, θ is the position angle, ξ is the dimensionless index along the bearing axis, *Pa* represents the ambient pressure, *c* represents the bearing radius clearance, *S*_*xx*_ and *S*_*yy*_ are the main stiffness values, *S*_*xy*_ and *S*_*yx*_ are the cross stiffness values, *D*_*xx*_ and *D*_*yy*_ refer to the main damping values, and *D*_*xy*_ and *D*_*yx*_ represent the cross damping values.

### 2.3 Diagnosis of system crack fault based on dynamic characteristics analysis of rotor

No matter it is a hybrid magnetic bearing-rotor system or an elastic foil gas bearing-rotor system, they both are important components of rotating machinery, so the rotating machinery shaft is prone to crack, which is the same case in the magnetic bearing-rotor system and gas bearing-rotor system, and has a great influence on the dynamic characteristics of the system. This paper takes the bearing-rotor system as the research object, introduces a CNN under deep learning, and applies the neural network model to the fault detection of the bearing-rotor system rotor.

CNN is one of the most widely used models in deep learning. In terms of structural composition, the input layer of CNN is mainly the input of correlation array [20]. The time domain signal of rotor vibration is used as input in this article, the convolutional layer containing several convolution kernels mainly completes the extraction of related data features [21], and the specific operation can be expressed as below.

$$x_{j}^{l}=f\left(\sum_{i}x_{i}^{l-1}*W_{ij}^{l}+b_{j}^{l}\right)$$ (5)

In the above equation, *f* corresponds to the activation function, $x_{j}^{l}$ represents the output of the *j*^*th*^ feature map in the *l*^*th*^ layer of CNN, $x_{i}^{l-1}$ represents the *i*^*th*^ feature map in the *l-1*^*th*^ layer of CNN, *W* refers to the connection weight, $b_{j}^{l}$ represents the deviation, and * corresponds to the convolution operation. This article chooses ReLU as the activation function. An important role of pooling layer under CNN is to reduce the number of parameters and redundant information in CNN [22]. In this article, the maximum pooling is selected for related operations; the main role of fully connected layer under CNN is to convert all learned features into a feature vector and to connect with the output layer [23]; and the output layer is to output the related features [24]. Softmax function is selected as the outputted classification label, which is specifically expressed as Eq (6).

$$p_{N}=\frac{\exp\left(x_{i}\right)}{\sum_{j=1}^{M}\exp\left(x_{j}\right)}$$ (6)

In the above equation, *N* corresponds to the number of labels, and *P*_*N*_ represents the probability value of the attributed label *N* in the input vector *x*_*i*_.

For the fault diagnosis and detection of the bearing-rotor system, four types of faults are considered, namely crack, misalignment, crack-misalignment coupling, and normal bearing-rotor system [25,26]. Related image recognition problems involved in this type of faults are relatively simple, so better classification can be achieved without too deep neural network structure. In addition, multiple stacking of convolution kernels can easily lead to data overfitting, so the number of convolutional layers in CNN is reduced appropriately with the premise of ensuring the accuracy of classification, so as to realize the recognition of different types of faults through Softmax classifier. The structure of the constructed CNN based on the fault diagnosis and classification of the bearing-rotor system is shown in Fig 3 below.

**Fig 3:** Structure for CNN based on fault diagnosis and classification of the bearing-rotor system.

Specifically, the CNN is mainly composed of three convolution layers and three pooling layers. The size of input layer is 5*1, and the size of pooling layer is 2*1. The Softmax classifier is used to achieve the output of the four types of failures in the bearing-rotor system. The determination of relevant parameters of the CNN model is analysed to find the most suitable CNN model for fault diagnosis of bearing rotor system.

### 2.4 Experiment setting

#### Analysis on dynamic characteristics of bearing-rotor system

The dynamic characteristics of the hybrid magnetic bearing-rotor system and the elastic foil gas bearing-rotor system are analysed with NI USB-6210 data acquisition instrument. The relevant parameters of the data acquisition instrument are shown in Table 1 below.

**Table 1:** Parameters of data acquisition instrument.

Parameter	Analogue input	Digital input	Digital output	Counter	Sensitivity of maximum voltage scope
Demonstration	16-lane	4-lane	4-lane	Two (32 bits)	91.6μV
Parameter	Maximum sampling rate	Resolution ratio	Maximum voltage scope	Accuracy of maximum voltage scope	
Demonstration	250 kS/s	16bits	-10-10 (V)	2.69mV	

On this basis, it analyses the stable and stationary state of hybrid magnetic bearing-rotor system and the changes in displacement and stiffness of the rotor caused by various loads in horizontal axis of the working wheel under different external load, so as to analyse and characterize the characteristics keeping dynamically stable state of rotor. What’s more, the changes in dynamic stiffness and damping in the elastic foil gas bearing-rotor system and the influencing effect of ambient pressure on dynamic characteristics of gas bearing-rotor system are analysed and characterized starting from the ambient pressure.

#### Experiment settings of fault detection for bearing-rotor system based on conventional neural network

On the basis of the above system experimental platform, the rotor vibration signals generated under several common fault types in the bearing-rotor system are acquired with the NI USB-6210 data acquisition instrument. The specific experimental implementation process is given as below. Regarding to the rotor crack faults in the bearing-rotor system, the cracked rotor is replaced according to the corresponding parameters of the cracks, and the misalignment faults caused by the coupling is simulated by padding the motor support part by 0.1mm. The rotating speed of the bearing-rotor system can be adjusted through regulation of the motor; specifically, to the vibration signals generated by the bearing-rotor system at different speeds in the range from 10Hz to 25Hz are collected with a data acquisition instrument and then transmitted to the signal acquisition system; the corresponding data acquisition frequency is 5kHz; and the signal data is collected cyclically by changing the generated fault type. Data signals at six different rotating speeds are selected for fusion processing, and the training and test data samples are formed in the means of repeating data sampling. The specific distribution of the rotor vibration time-domain signal after normalized fusion processing is shown in Fig 4 below. Each fault type contains 1,000 samples, of which each sample has 512 data points. Thus, the final data set is composed of 4,000 samples. Through random sampling, 70% is selected as the training set, and 30% as the test set.

**Fig 4:** Specific distribution of vibration time-domain signals of rotor.

In view of the classification of different types of faults in the bearing-rotor system, it is very necessary to determine the optimal CNN structure. In the CNN model, the size of the convolution kernel can affect the classification accuracy, while the batch size affects how fast the CNN model can process the amount of data. The larger the batch size, the faster the CNN model can process the amount of data. In addition, it can affect the convergence speed and accuracy. Based on the above experimental settings, the collected experimental signals are undertaken as the input of CNN to compare and analyse the accuracy of CNNs with different convolution kernel sizes and batch sizes in fault classification. The Adam optimization algorithm is adopted throughout the training process, and the learning rate is set to 0.001. Throughout the process of comparative analysis, the sizes of the convolution kernels are set to be the same in the second and third layer of the CNN. The fault classification effect of the CNN model is evaluated and analysed based on the changes in convolution kernel size, batch size, fault classification accuracy, and loss function of CNN, so as to determine the optimal structure of the CNN in the fault classification.

## 3. Results and discussion

### 3.1 Stability analysis of magnetic bearing-rotor system

Under the precondition that rotor is in a stable state, the displacement of the rotor in the hybrid magnetic bearing-rotor system and the X-direction stiffness change with the load are analysed when the working wheel in the bearing-rotor system is in the positive X direction and different external loads are applied, as shown in Fig 5 below Show.

**Fig 5:** Displacement and stiffness changes based on different external loads (In the figure, Wd represents the axial displacement change at the radial bearing on the working wheel side, Fd represents the axial displacement change at the radial bearing on the fan wheel side; Wr represents the stiffness change in X direction of the radial bearing on the working wheel side, and Fr represents the stiffness change in the X direction of the radial bearing on the fan wheel side).

Above figure illustrates that as the externally applied load continues to increase, the axial position of the radial bearing of the working wheel in the system deviates to the positive X direction. When the load increases from 0N to 40N, the offset changes from 0 to 22μm; at the same time, the axial position of the radial bearing of the fan wheel in the system deviates to the negative X direction, and the deviation changes from 0 to 16μm; as the applied load continues to increase, the offsets corresponding to the working wheel and the fan wheel increase continually, and the final maximum displacement offset is 135μm and 96μm, respectively. On the contrary, with the increase of the applied load, the stiffness values corresponding to the working wheel and the fan wheel in the system show decreasing trends, and finally fall to 35×10^5^N/m and 97.7×10^5^N/m, respectively.

The reason for such change is that the hybrid magnetic bearing-rotor system is realized by differential control. The control system adjusts the system current according to the rotor position offset signals detected by the sensor [27]. In addition, the material of the magnetic bearing is affected by the magnetic saturation performance, which brings a maximum value for the corresponding regulation current of the system. As the externally applied load continues to increase, the theoretically required system control current is reduced to zero in the positive X direction and the maximum control current in the negative X direction is the maximum value of the change in the bearing coil current to promote the rotor to return to the initial position. Under the synergistic effect of these variables and parameters, the stiffness of the system is reduced, and the displacement becomes larger.

### 3.2 Dynamic characteristics of elastic foil gas bearing-rotor system

Under different ambient pressures, the distribution and changes of the dynamic stiffness for the elastic foil gas bearing-rotor system are shown in Fig 6(A) and 6(B) below.

**Fig 6:** Distribution and changes of dynamic stiffness for gas bearing-rotor system: (a) S_xx_ and S_xy_; (b) S_yx_ and S_yy_.

The change of the system dynamic stiffness indicates that as the ambient pressure increases from 0.1 MPa to 0.5 MPa, the main dynamic stiffness S_xx_ and S_yy_ of the gas bearing show increasing trends, while the cross dynamic stiffness S_xy_ and S_yx_ show gradually decreasing trends; as the rotating speed of bearing continues to increase, the main dynamic stiffness of the gas bearing increases, while the cross dynamic stiffness shows a decreasing trend.

Under different ambient pressures, the distribution and changes of dynamic damping corresponding to the elastic foil gas bearing-rotor system are shown in Fig 7(a) and 7(b) below.

**Fig 7:** Distribution and changes of dynamic damping for gas bearing-rotor system: (a) D_xx_ and D_xy_; (b) D_yx_ and D_yy_.

The change of the system dynamic damping in the figure reveals that, the dynamic damping decreases with the increase of ambient pressure in the case of cross dynamic damping D_yx_ but increases with the increase of ambient pressure in all other conditions; with the increase of the rotating speed of the gas bearing, the dynamic damping of the gas bearing under other conditions decreases with the increase of the bearing rotating speed except the case in D_yx_.

When the corresponding length-diameter ratio of the gas bearing-rotor is 0.75, the eccentricity value is 0.6, and the vortex frequency value is 0.5, the distribution and changes of dynamic stiffness and dynamic damping for the gas bearing at various rotating speeds are analysed, as shown in Fig 8.

**Fig 8:** Distribution and changes of dynamic stiffness and dynamic damping for the gas bearing at various rotating speeds. Note: in the legend, S represents the dynamic stiffness, and D represents the dynamic damping.

After analysing the data changes in the figure, it can be found that with the continuous increase of the speed, the main stiffness S_xx_ and S_yy_ of the elastic foil gas bearing increase, the cross stiffness S_xy_ and S_yx_ change relatively slowly, the main damping D_xx_ and D_yy_ show decreasing trends, the cross damping D_yx_ becomes larger, and D_xy_ decreases.

Above results indicate that ambient pressure is beneficial to promote the improvement of elastic foil gas bearing performance, and the optimization effect of main stiffness and main damping based on dynamic characteristics analysis of elastic foil gas bearing is more significant. Thereby, it can be reasonably speculated that under the action of ambient pressure, the application fields of gas bearings under dynamic pressure can be expanded, so that the gas bearing can be equally applicable in other scenarios besides high-speed and light-load scenario. At the same time, the increase in ambient pressure can also improve the steady state of the gas bearing-rotor system at a smaller eccentricity. In short, increasing the ambient pressure of the gas bearing under certain precondition not only can promote the increase of the bearing capacity, but also can effectively enhance the stability optimization of the gas bearing-rotor system, thereby promoting the improvement and optimization of the dynamic characteristics of the system.

### 3.3 Parameter determination and fault classification efficiency of CNN model

Under different batch sizes, when the convolution kernel size of CNN model is 3*1, the classification accuracy and loss function changes for faults during the iteration process are shown in Fig 9 below.

**Fig 9:** Changes in classification accuracy and loss function when the convolution kernel size is 3*1 (in the figure, L represents the loss function, C represents the classification accuracy, and B represents the batch size).

As the number of iterations continues to increase, the classification and recognition accuracy of the final training set is close to 100%. When the batch size is 256, the classification and recognition accuracy of the testing set is 96.26% after 60 iterations. The loss function corresponding to the training function is close to zero at different numbers of iterations; the loss function corresponding to the testing set after 60 iterations is 0.07 when the batch size is 256, and with increase in number of iterations, it shows a decreasing trend as a whole.

Under different batch sizes, the changes in classification accuracy and loss function for faults during the iteration process are analysed when the CNN model convolution kernel size is 5*1, and the results are shown in Fig 10 below.

**Fig 10:** Changes in classification accuracy and loss function when the size of the convolution kernel is 5*1. Note: in the legend, L and C refers to the loss function and classification accuracy, respectively.

Under different numbers of iterations, the classification and recognition accuracy of the training set under different batch sizes is close to 100%. When the batch size is 32 and 64, the classification and recognition accuracy of the testing set is not very stable. When the batch size is 128 and 256, the final classification and recognition accuracy is 98.24% and 99.834%, respectively; and the classification accuracy is relatively stable as a whole. The loss function corresponding to the training set is also close to zero, the loss function changes greatly when the batch size is 32 and 64, and the final corresponding loss function are 0.05 and 0.03 when the batch size is 128 and 256, respectively, so the loss function shows a downward trend in general.

Under different batch sizes, the changes in classification accuracy and loss function for faults during the iteration process are analysed when the CNN model convolution kernel size is 7*1, as shown in Fig 11 below.

**Fig 11:** Changes in classification accuracy and loss function when the convolution kernel size is 7*1. Note: in the legend, L and C refers to the loss function and classification accuracy, respectively.

When the batch size is 32 and 64, the classification and recognition accuracy corresponding to the testing set fluctuates greatly and the overall value is small. When the batch size is 128 and 256, the classification and recognition accuracy corresponding to the testing set is relatively high and stable during the whole iteration. The loss function of the testing set is unstable under the premise that the batch size is 32 and 64, it shows a decreasing trend under the premise that the batch size is 128 and 256.

Based on the above analysis, it can be concluded that when the size of the convolution kernel in CNN is 7*1 and the batch size is 128, the CNN model constructed in this article shows good convergence performance in the classification and recognition accuracy and loss function during the entire iteration process. At the same time, the classification and recognition accuracy corresponding to the testing set and training set is the best, and the loss function is relatively small. Therefore, the final structure of the CNN model is determined as that the size of convolution kernel in the first layer is 32*1, the size of convolution kernel in the next two layers is 7*1, and the size in the pooling layer is 2*1.

## 4. Conclusion

The dynamic characteristics of the hybrid electromagnetic bearing-rotor system is analyzed based on the rotor displacement and stiffness. It is found that the acceleration of the electromagnetic bearing speed increases the displacement of the rotor and decreases the stiffness. The increased environmental pressure plays a positive role in the optimization of the gas bearing-rotor system. A convolution kernel with a size of 7*1 and a batch size of 128 shows the best performance in the classification and detection of faults. This research exerts an active role in promoting the study and development of the dynamic characteristics of the electromagnetic bearing-rotor system. However, identification of cracks is not analyzed specifically. The actual application of the CNN model in fault diagnosis has not been involved. In addition, the relevant influencing factors of analyzing the dynamic characteristics of bearing-rotor system have not been expanded for detailed analysis. In the future research, the identification of cracks will be added, and more influence factors will be introduced to analyze the dynamic characteristics of the bearing-rotor system.

## Supporting information

S1 Data (XLSX)
